# Conservative management of avascular necrosis of the metacarpal head: A case report and brief review

This article has been retracted.

**DOI:** 10.1097/MD.0000000000026083

**Published:** 2021-05-21

**Authors:** Xiao-Lei Fan, Wen-Tao Wang, Jian Wang, Yi Liao, Rui Xiao, Yi-He Hu

**Affiliations:** a Department of Orthopaedic Surgery, Xiangya Hospital, Central South University, Changsha; b Department of Medical Imaging Center; c Department of Orthopaedic Surgery, Karamay Central Hospital, Karamay, China.

**Keywords:** avascular necrosis, conservative treatment, dieterich's disease, metacarpal head, osteonecrosis

## Abstract

**Rationale:**

Avascular necrosis (AVN) of the metacarpal head is rare, and there is no clear consensus on treatment. The main aim of this study was to discuss the possible pathologic-mechanics of its development, epidemiology, radiographic features, and outcome after conservative treatment.

**Patient concerns:**

A 14-year-old male with a history of fractures in little finger complained of right-hand pain with a limited range of motion for 1 month. Diagnosis: Imaging examination confirmed the diagnosis of AVN in the long metacarpal finger and ring finger.

**Interventions:**

The patient was treated using non-surgical management, such as splint immobilization, non-steroidal anti-inflammatory drugs, and physiotherapy.

**Outcomes:**

At the last follow-up 26 months later, the patient was in complete remission with no residual symptoms. Magnetic resonance imaging (MRI) confirmed excellent remodeling and regeneration in the metacarpal head.

**Lessons:**

Metacarpal head necrosis typically occurs in adolescent patients with a history of trauma. Conservative treatment may sometimes have an excellent prognosis.

## 1 Introduction

Avascular necrosis (AVN) of the metacarpal head is a rare disease. The earliest description of the disease was reported by Mauclaire (1927), but it was referred to as dieterich disease with an unknown etiology.^[1–3]^ A comprehensive literature review indicates that there are few studies which have reported about AVN of the metacarpal head, most of which are case reports. Presently, there are about 50 cases of AVN of the metacarpal head which have been reported in the literature.^[3]^ The studies have reported that the patients’ age range between 6 and 82 years, with teenagers being predominantly affected by the disease.^[4,5]^ Wright and Dell^[1]^ reported that occurrence of the disease is slightly more predominant in men than in women, with the male-to-female ratio being 3:2. Despite dieterich's disease being observed in all metacarpals, it is mostly common in the middle finger and most rarely found in the thumb.^[1,3]^

The clinical symptoms vary in severity, ranging from asymptomatic to pain, swelling, and limited movement of the metacarpophalangeal joint.^[6,7]^ The disease is characterized by the lack of a uniform diagnostic criteria and treatment method. Moreover, plain radiographs may report as normal in the early stage of AVN. Magnetic resonance imaging (MRI) is the most sensitive tool for the diagnosis of AVN of the metacarpal,^[7,8]^ and bone scintigraphy can be helpful in discovering AVN and screening for other bone lesions.^[9,10]^ However, there is no clear consensus on the best treatment strategy due to the rarity of the condition. Therefore, management of hand AVN can be a challenging problem with a variety of procedures being described for its treatment. Most of the treatment methods are surgical, and there are very few cases of conservative treatment.

## 2 Case presentation

The patient in this study was a 14-year-old right-hand dominant male, presenting with the main complaint of pain and swelling in the right little finger. The symptoms were presented after he punched a wall. Swelling and tenderness were observed on the fifth metacarpal after examination of his right hand. In addition, radiographs showed a nondisplaced metacarpal neck fracture on his right little finger (Fig. 1a). The finger was put in a cast for 1 month and the patient was then instructed to begin active motion exercises after removal of the cast.

**Figure 1:** (A) Oblique radiograph showing a metacarpal neck fracture on the right little finger. (B) Anteroposterior radiograph demonstrating subchondral collapse and sclerotic changes in the long finger (red arrow) and ring finger (yellow arrow) metacarpal head.

After 5 months, he noted gradual pain in the long finger and ring finger metacarpophalangeal (MCP) joint. The patient came to our department again due to the persisting discomfort, reduced grip strength, and limited extension of the MCP joint. He exhibited mild swelling and tenderness to palpation at the long finger and ringer finger MCP joint. Moreover, active and passive motion was painful, and the Visual Analogue Scale score for pain was 5. There was full active flexion, but the extension was limited to 30° and was associated with pain. The obtained X-rays images indicated subchondral collapse and sclerotic changes in the metacarpal head (Fig. 1b). The serological investigation for inflammatory markers was normal, while CT scanning demonstrated cystic, osteochondral defect, and sclerotic changes (Fig. 2). The patient had no history of any predisposing systemic illnesses such as autoimmune disease or steroid use. Thus, he was diagnosed with AVN of the metacarpal head or dieterich's disease based on the clinical and radiographic findings.

**Figure 2:** Sagittal images of computed tomography indicating cystic, osteochondral defect, and sclerotic changes in the long finger (red arrow, A, B) and ring finger (yellow arrow, C, D) metacarpal head.

Conservative management was initially offered due to the young age and spontaneous remodeling. He was then treated using splint immobilization for 3 weeks in combination with nonsteroidal anti-inflammatory drug and physiotherapy. The patient was also advised to use his hand as normally as possible within the limits of pain. He experienced gradual relieving of the pain in the region of the MCP joint after 4 months and there were no obvious restrictions of activities of daily living. In addition, conservative treatment and follow-up were recommended although there was no significant change in the imaging examination.

The follow up examination done 26 months after fracture indicated that there was a painless full range of active motion. Radiographs showed remodeling of the long finger and ring finger metacarpal head (Fig. 3). Moreover, there were no radiographic signs of hyperostosis, osteosclerosis, or osteoarthritis. MRI indicated no bone marrow edema, joint effusion, or subchondral fractures within the affected metacarpal head (Fig. 4). In addition, the image examinations revealed that further remodeling of the MCP joint had occurred. The patient's cosmetic result and range of motion were excellent at the last follow-up (Fig. 5), and the grip strength and range of motion of the affected MCP joints were almost equal to the contralateral. Furthermore, the Visual Analogue Scale score for pain was zero, and no residual pain was left. Therefore, no further specific treatment was recommended.

**Figure 3:** Anteroposterior (A) and oblique (B) radiographs demonstrating remodeling of the long finger (red arrow) and ring finger (yellow arrow) metacarpal head.

**Figure 4:** T1-weighted sagittal (A, C) and T2-weighted coronal (B) images showing no bone marrow edema, joint effusion, or subchondral fractures within the long finger (red arrow) and ring finger (yellow arrow) metacarpal head.

**Figure 5:** (A, B) Function image showing full flexion of the metacarpophalangeal (MCP) joint.

## 3 Discussion and conclusion

AVN of the metacarpal head is a rare disease and its etiology has not yet been elucidated. It has been named idiopathic because it can occur without any obvious cause.^[11–14]^ Although it is commonly idiopathic, as with other aseptic bone necrosis, a connection to steroid intake is discussed in dietrich's disease.^[1,15]^ Moreover, comorbidities like system lupus erythematosus,^[1,16]^ Freiberg disease,^[9]^ and juvenile dermatomyositis^[17]^ have been described. Some studies have also reported its association with trauma and anatomic variations in the blood supply to the metacarpal head.^[2,3,7]^ Adolescents make up a large proportion of the cases, with more than 50% of the reported patients being under the age of 20.^[3]^ In addition to individuals with definite steroid use, most of the patients have a history of trauma.^[3,7,18,19]^

Wright and Dell^[1]^ conducted a metacarpal vascular anatomy study which reported an absence of large nutrient vessels in 35% of the specimens, which may place distal metacarpal epiphyses at risk for AVN development. In addition, no vessels were observed across the physeal scar. The metacarpal heads solely relied on small pericapsular circumferential arterioles because they lacked significant intraosseous vascularization. Therefore, anatomic variations in the blood supply to the metacarpal head may be a potential factor rendering some individuals at an increased risk for osteonecrosis.^[1]^

The prominent position of the metacarpal head may frequently sustain occult trauma without notice. Blunt trauma to the metacarpal head area can result in an occult microfracture with metacarpophalangeal joint effusion, which may compress the periosteal blood vessels to the distal epiphysis and thus delay venous return.^[1,8,14]^ In the face of a traumatic effusion, a tamponade effect of these vessels may result in avascularity of the distal epiphysis with concomitant bone and cartilage necrosis and collapse. Gannon et al,^[8]^ speculated that the chronic and repetitive loading of the metacarpal heads may have led to the avascular changes. In another study, digital subtraction angiography showed venous pooling in the affected metacarpal heads.^[14]^ This finding suggests that there might be a delay in venous return, thereby resulting in increased intramedullary pressure and hypoxia. On the other hand, the increased bone marrow pressure might have caused bone marrow edema and transient osteoporosis, thereby resulting in the collapse of the metacarpal head.^[14]^ Sagar^[7]^ reported 2 pediatric cases of AVN of the fourth metacarpal head, which was secondary to indirect trauma. One of the patients also suffered a fifth metacarpal neck fracture before AVN, similar to our case.

Clinical symptoms and imaging examinations are the main tools for the diagnosis of osteonecrosis. A high degree of suspicion is required, especially if the patient has a preceding history of trauma. Conventional X-rays show characteristic changes with disturbance of the trabecular pattern, flattening, and sclerosis.^[20]^ The characteristic findings of AVN using MRI include: T1-weighted images indicated diminished signal intensity within a background of the bright signal of fatty marrow, while T2-weighted sequences displayed a distinctive pattern designated the double-line sign.^[8]^ In addition, bone scintigraphy can be helpful in discovering increased uptake at the MCP joint in the early stages.^[10]^ The introduction of bone scintigraphy techniques can help in early diagnosis and improve treatment outcomes.

Currently, there is no standard treatment for this disease. Majority of the reported cases were initially handled using non-surgical methods. Rest, immobilization, and use of non-steroidal anti-inflammatory medications may be sufficient to control the symptoms. Moreover, conservative treatment has also been reported as being successful.^[2,3,21]^ However, the duration of the course of nonsurgical management was ambiguous. In most cases, the nonsurgical management was followed up for 3 months.^[6]^ Similarly, another study offered nonsurgical management to all patients for 3 to 6 months. The obtained results indicated that 2 patients had full active range of motion, and the pain symptoms were improved.^[3]^ The duration of conservative treatment should be longer for adolescents, especially those with multiple lesions. Children who are still experiencing bone remodeling and growth may experience spontaneous improvement in AVN in non–weight-bearing areas. A previous study reported that the metacarpal head of a steroid-treated nephrotic syndrome patient was completely regenerated after AVN, although no treatment was given.^[4]^ In another study, the obtained radiographs revealed spontaneous remodeling of the MCP joint in a case of metacarpal necrosis in a 14-year-old boy.^[2]^ Therefore, given the potential for bone remodeling, patients with pediatric metacarpal AVN may recover after receiving conservative treatment.^[2,12,17]^

Many articles have described the surgical management of AVN of the metacarpal head. In most cases, the decision to proceed with surgery was made after failure of conservative treatment. Bone curettage and cancellous bone grafting ^[3,6,13]^, flexion osteotomy,^[20]^ metatarsal transplantation,^[22]^ costal osteochondral autograft,^[14,23]^ osteochondral autograft transplantation surgery,^[18,24]^ arthroplasty,^[25,26]^ and arthrodesis^[27]^ have been performed in individual cases. The type of surgery depends on the condition of the damaged cartilage layer. Subchondral curettage and cancellous bone grafting give excellent results in instances where the cartilage is still good,^[28]^ while other joints preserving surgery techniques may be necessary in instances where the cartilage is destroyed.

Curettage and cancellous bone graft are one of the most widely used surgical methods. This method can preserve the intact cartilage layer and provide it with a solid underlying bony base.^[3,6,13]^ Therefore, curettage and cancellous bone grafting is a good choice for early-stage patients with an intact articular surface. In addition, osteochondral plug harvesting from the none-weight bearing articular surface of the knee, transferring, and pressing-fit to resurface a focal metacarpal head lesions is an effective method. A special osteochondral harvester is usually required, and thus there may be a risk of damaging the growth plate.^[18,24]^ Arthrodesis or joint replacement should be considered as salvage operations when cartilage erosion is severe or joint surfaces collapse with persistent symptoms. Almost all the operating cases have reported excellent results. However, the long-term prognosis is unknown and instability or other complications of the MCP joint may require revision.

Many scholars believe that patients undergoing conservative treatment may be at an increased risk of early arthritic involvement of the MCP joint in the future.^[6,8,20,23]^ However, even surgical treatment cannot completely avoid this risk. Therefore, conservative treatment can be applied as long as there are no pain symptoms, and the function is normal. Surgery should only be considered if the symptoms return and become refractory to conservative measures for several years.

This study reports a typical case that will enlarge the existing sample size and provide further conservative treatment information for dietrich's disease. Although AVN of the metacarpal head is rare, more attention should be paid to the adolescent with a preceding history of trauma. MRI is the most sensitive tool for the diagnosis of AVN of metacarpal head, besides it can evaluate the remodeling and regeneration of metacarpal head.

## Acknowledgments

We thank the patients involved in the study. We want to thank Xiao-Huan Jia for technological support.

## Author contributions

**Conceptualization:** Rui Xiao.

**Data curation:** Xiao-Lei Fan, Jian Wang.

**Formal analysis:** Xiao-Lei Fan, Wen-Tao Wang.

**Project administration:** Yi-He Hu.

**Supervision:** Yi Liao, Rui Xiao.

**Writing – original draft:** Xiao-Lei Fan, Wen-Tao Wang.

**Writing – review & editing:** Rui Xiao, Yi-He Hu.
